# Bis(2-eth­oxy-6-formyl­phenolato-κ^2^ *O* ^1^,*O* ^6^)nickel(II)

**DOI:** 10.1107/S160053680800809X

**Published:** 2008-03-29

**Authors:** Zhen-Quan Han

**Affiliations:** a Applied Technical College, Qiqihar University, Qiqihar 161006, People’s Republic of China

## Abstract

The title compound, [Ni(C_9_H_9_O_3_)_2_], was synthesized by the reaction of 3-ethoxy­salicylaldehyde with nickel(II) nitrate in methanol solution. The asymmetric unit onsists of two half-molecules; each Ni atom lies on a centre of symmetry. The  Ni^II^ ions are coordinated by four O atoms from two deprotonated 3-ethoxy­salicylaldehyde ligands in a slightly distorted square-planar coordination environment.

## Related literature

For related literature, see: Carlsson *et al.* (2004 ▶); Li & Chen (2006 ▶); Mounts & Fernando (1974 ▶); Volkmer *et al.* (1996 ▶).

## Experimental

### 

#### Crystal data

[Ni(C_9_H_9_O_3_)_2_]
*M* *_r_* = 389.03
Triclinic,
*a* = 8.448 (2) Å
*b* = 10.123 (2) Å
*c* = 11.919 (3) Å
α = 111.175 (2)°
β = 97.377 (2)°
γ = 102.431 (3)°
*V* = 904.1 (4) Å^3^
*Z* = 2
Mo *K*α radiation
μ = 1.10 mm^−1^
*T* = 298 (2) K
0.32 × 0.32 × 0.30 mm

#### Data collection

Bruker SMART CCD area-detector diffractometer
Absorption correction: multi-scan (*SADABS*; Sheldrick, 1996 ▶) *T*_min_ = 0.719, *T*_max_ = 0.733
5465 measured reflections
3993 independent reflections
3187 reflections with *I* > 2σ(*I*)
*R*_int_ = 0.013

#### Refinement

*R*[*F* ^2^ > 2σ(*F* ^2^)] = 0.041
*wR*(*F* ^2^) = 0.116
*S* = 1.02
3993 reflections
231 parameters
H-atom parameters constrained
Δρ_max_ = 0.65 e Å^−3^
Δρ_min_ = −0.66 e Å^−3^

### 

Data collection: *SMART* (Bruker, 1998 ▶); cell refinement: *SAINT* (Bruker, 1998 ▶); data reduction: *SAINT*; program(s) used to solve structure: *SHELXS97* (Sheldrick, 2008 ▶); program(s) used to refine structure: *SHELXL97* (Sheldrick, 2008 ▶); molecular graphics: *SHELXTL* (Sheldrick, 2008 ▶); software used to prepare material for publication: *SHELXTL*.

## Supplementary Material

Crystal structure: contains datablocks global, I. DOI: 10.1107/S160053680800809X/lh2604sup1.cif

Structure factors: contains datablocks I. DOI: 10.1107/S160053680800809X/lh2604Isup2.hkl

Additional supplementary materials:  crystallographic information; 3D view; checkCIF report

## Figures and Tables

**Table:** 

Ni1—O5	1.837 (2)
Ni1—O4	1.852 (2)
Ni2—O1	1.843 (2)
Ni2—O2	1.851 (2)

**Table:** 

O5—Ni1—O5^i^	180
O5—Ni1—O4	94.16 (9)
O5^i^—Ni1—O4	85.84 (9)
O4—Ni1—O4^i^	180
O1—Ni2—O1^ii^	180
O1—Ni2—O2	93.70 (9)
O1^ii^—Ni2—O2	86.30 (9)
O2^ii^—Ni2—O2	180

Symmetry codes: (i) ; (ii) .

## supplementary crystallographic information

### Comment

The authors interest in nickel(II) complexes arises from the fact that Ni(II) is the active center of the urease enzyme (Carlsson *et al.*, 2004; Volkmer *et al.*, 1996). The author reports herein the crystal structure of the title nickel(II) complex.

In the asymmetric unit of the title compound, there are two independent complex (Fig. 1). Each Ni^II^ ion lies on an inversion center and is coordinated by four O atoms from two deprotonated 3-ethoxysalicylaldehyde ligands. The coordinate bond values (Table 1) in each molecule are comparable to each other between the two independent complex molecules. The structure is similar to other nickel(II) complexes derived from the derivatives of salicylaldehyde (Li & Chen, 2006; Mounts & Fernando, 1974).

### Experimental

All chemicals were of AR grade. 3-Ethoxysalicylaldehyde (33.2 mg, 0.2 mmol) and nickel(II) nitrate hexahydrate (29.0 mg, 0.1 mmol) were refluxed for 30 min in 10 ml methanol solution. The mixture was cooled to room temperature and filtered. Keeping the filtrate in air for a week, yielded red block crystals suitable for X-ray analysis.

### Refinement

H atoms were placed in idealized positions and constrained to ride on their parent atoms with C–H distances in the range 0.93–0.97 Å, and with *U*_iso_(H) set at 1.2*U*_eq_(C) and 1.5*U*_eq_(methyl C). Although no significant density was located in the solvent accessible VOIDS of 47.00 Å^3^, these might be able to accommodate disordered water molecules.

### Crystal data

**Table:**

[Ni(C_9_H_9_O_3_)_2_]	*Z* = 2
*M**_r_* = 389.03	*F*_000_ = 404
Triclinic, *P*1	*D*_x_ = 1.429 Mg m^−^^3^
Hall symbol: -P 1	Mo *K*α radiation λ = 0.71073 Å
*a* = 8.448 (2) Å	Cell parameters from 2386 reflections
*b* = 10.123 (2) Å	θ = 2.2–27.9º
*c* = 11.919 (3) Å	µ = 1.10 mm^−^^1^
α = 111.175 (2)º	*T* = 298 (2) K
β = 97.377 (2)º	Block, red
γ = 102.431 (3)º	0.32 × 0.32 × 0.30 mm
*V* = 904.1 (4) Å^3^	

### Data collection

**Table:**

Bruker SMART CCD area-detector diffractometer	3993 independent reflections
Radiation source: fine-focus sealed tube	3187 reflections with *I* > 2σ(*I*)
Monochromator: graphite	*R*_int_ = 0.013
*T* = 298(2) K	θ_max_ = 27.5º
ω scans	θ_min_ = 2.3º
Absorption correction: multi-scan(SADABS; Sheldrick, 1996)	*h* = −10→8
*T*_min_ = 0.719, *T*_max_ = 0.733	*k* = −13→13
5465 measured reflections	*l* = −11→15

### Refinement

**Table:**

Refinement on *F*^2^	Secondary atom site location: difference Fourier map
Least-squares matrix: full	Hydrogen site location: inferred from neighbouring sites
*R*[*F*^2^ > 2σ(*F*^2^)] = 0.041	H-atom parameters constrained
*wR*(*F*^2^) = 0.116	*w* = 1/[σ^2^(*F*_o_^2^) + (0.0596*P*)^2^ + 0.672*P*] where *P* = (*F*_o_^2^ + 2*F*_c_^2^)/3
*S* = 1.02	(Δ/σ)_max_ < 0.001
3993 reflections	Δρ_max_ = 0.65 e Å^−^^3^
231 parameters	Δρ_min_ = −0.66 e Å^−^^3^
Primary atom site location: structure-invariant direct methods	Extinction correction: none

### Special details

**Table:**

Geometry. All e.s.d.'s (except the e.s.d. in the dihedral angle between two l.s. planes) are estimated using the full covariance matrix. The cell e.s.d.'s are taken into account individually in the estimation of e.s.d.'s in distances, angles and torsion angles; correlations between e.s.d.'s in cell parameters are only used when they are defined by crystal symmetry. An approximate (isotropic) treatment of cell e.s.d.'s is used for estimating e.s.d.'s involving l.s. planes.
Refinement. Refinement of *F*^2^ against ALL reflections. The weighted *R*-factor *wR* and goodness of fit *S* are based on *F*^2^, conventional *R*-factors *R* are based on *F*, with *F* set to zero for negative *F*^2^. The threshold expression of *F*^2^ > σ(*F*^2^) is used only for calculating *R*-factors(gt) *etc*. and is not relevant to the choice of reflections for refinement. *R*-factors based on *F*^2^ are statistically about twice as large as those based on *F*, and *R*- factors based on ALL data will be even larger.

### Fractional atomic coordinates and isotropic or equivalent isotropic displacement parameters (Å^2^)

**Table:**

	*x*	*y*	*z*	*U*_iso_*/*U*_eq_	
Ni1	0.0000	0.5000	0.0000	0.02805 (13)	
Ni2	0.0000	0.0000	0.0000	0.02920 (14)	
O1	0.0505 (2)	−0.0121 (2)	0.15045 (16)	0.0363 (4)	
O2	−0.0576 (3)	0.1741 (2)	0.0663 (2)	0.0506 (5)	
O3	0.1596 (3)	−0.0689 (2)	0.33683 (18)	0.0484 (5)	
O4	0.0529 (3)	0.3494 (3)	−0.1190 (2)	0.0513 (5)	
O5	0.1989 (2)	0.63719 (19)	0.02863 (17)	0.0350 (4)	
O6	0.4541 (3)	0.8659 (2)	0.1053 (2)	0.0552 (6)	
C1	0.3232 (3)	0.4873 (3)	−0.1220 (3)	0.0366 (6)	
C2	0.3219 (3)	0.6192 (3)	−0.0278 (2)	0.0328 (5)	
C3	0.4641 (3)	0.7438 (3)	0.0107 (3)	0.0416 (7)	
C4	0.5959 (4)	0.7345 (4)	−0.0462 (3)	0.0534 (8)	
H4	0.6872	0.8170	−0.0214	0.064*	
C5	0.5940 (4)	0.6031 (4)	−0.1404 (3)	0.0583 (9)	
H5	0.6837	0.5983	−0.1779	0.070*	
C6	0.4608 (4)	0.4814 (4)	−0.1777 (3)	0.0508 (8)	
H6	0.4606	0.3938	−0.2403	0.061*	
C7	0.1866 (3)	0.3570 (3)	−0.1613 (3)	0.0387 (6)	
H7	0.1946	0.2713	−0.2220	0.046*	
C8	0.5934 (4)	0.9930 (4)	0.1562 (4)	0.0630 (10)	
H8A	0.6162	1.0304	0.0939	0.076*	
H8B	0.6910	0.9687	0.1859	0.076*	
C9	0.5528 (5)	1.1062 (5)	0.2603 (4)	0.0745 (11)	
H9A	0.4523	1.1251	0.2308	0.112*	
H9B	0.6424	1.1959	0.2933	0.112*	
H9C	0.5375	1.0706	0.3238	0.112*	
C10	0.0426 (4)	0.2306 (3)	0.2817 (3)	0.0403 (6)	
C11	0.0741 (3)	0.0937 (3)	0.2595 (2)	0.0344 (6)	
C12	0.1373 (4)	0.0681 (3)	0.3646 (3)	0.0408 (6)	
C13	0.1716 (5)	0.1762 (4)	0.4812 (3)	0.0603 (9)	
H13	0.2143	0.1582	0.5484	0.072*	
C14	0.1433 (6)	0.3135 (4)	0.5010 (3)	0.0737 (12)	
H14	0.1689	0.3866	0.5806	0.088*	
C15	0.0782 (5)	0.3389 (4)	0.4027 (3)	0.0604 (10)	
H15	0.0571	0.4292	0.4158	0.073*	
C16	−0.0311 (4)	0.2596 (3)	0.1806 (3)	0.0390 (6)	
H16	−0.0617	0.3467	0.1996	0.047*	
C17	0.2484 (5)	−0.0970 (4)	0.4322 (3)	0.0552 (8)	
H17A	0.1831	−0.0992	0.4930	0.066*	
H17B	0.3528	−0.0202	0.4733	0.066*	
C18	0.2804 (6)	−0.2441 (5)	0.3720 (4)	0.0832 (14)	
H18A	0.1769	−0.3208	0.3414	0.125*	
H18B	0.3527	−0.2606	0.4315	0.125*	
H18C	0.3322	−0.2449	0.3047	0.125*	

### Atomic displacement parameters (Å^2^)

**Table:**

	*U*^11^	*U*^22^	*U*^33^	*U*^12^	*U*^13^	*U*^23^
Ni1	0.0239 (2)	0.0277 (2)	0.0327 (2)	0.00622 (17)	0.00861 (17)	0.01208 (19)
Ni2	0.0308 (2)	0.0285 (2)	0.0283 (2)	0.00865 (18)	0.00732 (18)	0.01098 (18)
O1	0.0484 (11)	0.0311 (9)	0.0290 (9)	0.0129 (8)	0.0067 (8)	0.0113 (8)
O2	0.0517 (13)	0.0484 (12)	0.0514 (13)	0.0158 (10)	0.0160 (10)	0.0173 (10)
O3	0.0639 (14)	0.0438 (12)	0.0361 (10)	0.0201 (10)	0.0001 (10)	0.0152 (9)
O4	0.0470 (12)	0.0502 (13)	0.0537 (13)	0.0132 (10)	0.0147 (10)	0.0164 (11)
O5	0.0277 (9)	0.0310 (9)	0.0459 (11)	0.0057 (7)	0.0132 (8)	0.0149 (8)
O6	0.0374 (11)	0.0432 (12)	0.0731 (16)	−0.0024 (9)	0.0148 (11)	0.0170 (11)
C1	0.0303 (13)	0.0484 (16)	0.0388 (14)	0.0144 (12)	0.0129 (11)	0.0225 (12)
C2	0.0246 (12)	0.0412 (14)	0.0404 (14)	0.0104 (10)	0.0093 (10)	0.0238 (12)
C3	0.0300 (13)	0.0469 (17)	0.0530 (18)	0.0070 (12)	0.0110 (12)	0.0272 (15)
C4	0.0316 (15)	0.061 (2)	0.072 (2)	0.0021 (14)	0.0163 (15)	0.0362 (18)
C5	0.0380 (17)	0.079 (3)	0.069 (2)	0.0179 (17)	0.0286 (16)	0.036 (2)
C6	0.0414 (16)	0.065 (2)	0.0521 (18)	0.0205 (15)	0.0228 (14)	0.0239 (16)
C7	0.0367 (14)	0.0426 (15)	0.0386 (14)	0.0161 (12)	0.0154 (12)	0.0132 (12)
C8	0.0436 (18)	0.055 (2)	0.076 (3)	−0.0064 (16)	0.0034 (17)	0.0253 (19)
C9	0.073 (3)	0.060 (2)	0.064 (2)	−0.008 (2)	0.005 (2)	0.0134 (19)
C10	0.0472 (16)	0.0387 (15)	0.0354 (14)	0.0168 (13)	0.0131 (12)	0.0114 (12)
C11	0.0318 (13)	0.0374 (14)	0.0314 (13)	0.0086 (11)	0.0091 (10)	0.0110 (11)
C12	0.0423 (15)	0.0421 (15)	0.0341 (14)	0.0127 (12)	0.0064 (12)	0.0115 (12)
C13	0.084 (3)	0.064 (2)	0.0297 (15)	0.030 (2)	0.0049 (16)	0.0120 (15)
C14	0.114 (3)	0.064 (2)	0.0347 (17)	0.041 (2)	0.0089 (19)	0.0036 (16)
C15	0.093 (3)	0.0484 (19)	0.0391 (17)	0.0340 (19)	0.0151 (17)	0.0092 (14)
C16	0.0474 (16)	0.0345 (14)	0.0392 (15)	0.0176 (12)	0.0166 (12)	0.0139 (12)
C17	0.062 (2)	0.065 (2)	0.0424 (17)	0.0247 (17)	0.0015 (15)	0.0249 (16)
C18	0.118 (4)	0.077 (3)	0.062 (2)	0.057 (3)	0.000 (2)	0.027 (2)

### Geometric parameters (Å, °)

**Table:**

Ni1—O5	1.837 (2)	C6—H6	0.9300
Ni1—O5^i^	1.837 (2)	C7—H7	0.9300
Ni1—O4	1.852 (2)	C8—C9	1.491 (5)
Ni1—O4^i^	1.852 (2)	C8—H8A	0.9700
Ni2—O1	1.843 (2)	C8—H8B	0.9700
Ni2—O1^ii^	1.843 (2)	C9—H9A	0.9600
Ni2—O2^ii^	1.851 (2)	C9—H9B	0.9600
Ni2—O2	1.851 (2)	C9—H9C	0.9600
O1—C11	1.309 (3)	C10—C11	1.405 (4)
O2—C16	1.282 (3)	C10—C15	1.406 (4)
O3—C12	1.365 (3)	C10—C16	1.438 (4)
O3—C17	1.429 (3)	C11—C12	1.430 (4)
O4—C7	1.294 (3)	C12—C13	1.369 (4)
O5—C2	1.319 (3)	C13—C14	1.402 (5)
O6—C3	1.367 (4)	C13—H13	0.9300
O6—C8	1.417 (4)	C14—C15	1.362 (5)
C1—C2	1.404 (4)	C14—H14	0.9300
C1—C6	1.412 (4)	C15—H15	0.9300
C1—C7	1.432 (4)	C16—H16	0.9300
C2—C3	1.426 (4)	C17—C18	1.502 (5)
C3—C4	1.380 (4)	C17—H17A	0.9700
C4—C5	1.391 (5)	C17—H17B	0.9700
C4—H4	0.9300	C18—H18A	0.9600
C5—C6	1.364 (5)	C18—H18B	0.9600
C5—H5	0.9300	C18—H18C	0.9600
			
O5—Ni1—O5^i^	180	O6—C8—H8B	110.2
O5—Ni1—O4	94.16 (9)	C9—C8—H8B	110.2
O5^i^—Ni1—O4	85.84 (9)	H8A—C8—H8B	108.5
O5—Ni1—O4^i^	85.84 (9)	C8—C9—H9A	109.5
O5^i^—Ni1—O4^i^	94.16 (9)	C8—C9—H9B	109.5
O4—Ni1—O4^i^	180	H9A—C9—H9B	109.5
O1—Ni2—O1^ii^	180	C8—C9—H9C	109.5
O1—Ni2—O2^ii^	86.30 (9)	H9A—C9—H9C	109.5
O1^ii^—Ni2—O2^ii^	93.70 (9)	H9B—C9—H9C	109.5
O1—Ni2—O2	93.70 (9)	C11—C10—C15	120.7 (3)
O1^ii^—Ni2—O2	86.30 (9)	C11—C10—C16	120.0 (2)
O2^ii^—Ni2—O2	180	C15—C10—C16	119.3 (3)
C11—O1—Ni2	126.59 (17)	O1—C11—C10	125.3 (2)
C16—O2—Ni2	127.6 (2)	O1—C11—C12	117.4 (2)
C12—O3—C17	118.6 (2)	C10—C11—C12	117.3 (2)
C7—O4—Ni1	127.6 (2)	O3—C12—C13	125.1 (3)
C2—O5—Ni1	127.62 (17)	O3—C12—C11	114.3 (2)
C3—O6—C8	118.6 (3)	C13—C12—C11	120.5 (3)
C2—C1—C6	120.1 (3)	C12—C13—C14	121.2 (3)
C2—C1—C7	120.5 (2)	C12—C13—H13	119.4
C6—C1—C7	119.4 (3)	C14—C13—H13	119.4
O5—C2—C1	125.0 (2)	C15—C14—C13	119.4 (3)
O5—C2—C3	117.0 (2)	C15—C14—H14	120.3
C1—C2—C3	118.0 (2)	C13—C14—H14	120.3
O6—C3—C4	125.7 (3)	C14—C15—C10	120.9 (3)
O6—C3—C2	114.0 (2)	C14—C15—H15	119.6
C4—C3—C2	120.3 (3)	C10—C15—H15	119.6
C3—C4—C5	120.8 (3)	O2—C16—C10	124.7 (3)
C3—C4—H4	119.6	O2—C16—H16	117.6
C5—C4—H4	119.6	C10—C16—H16	117.6
C6—C5—C4	120.2 (3)	O3—C17—C18	107.2 (3)
C6—C5—H5	119.9	O3—C17—H17A	110.3
C4—C5—H5	119.9	C18—C17—H17A	110.3
C5—C6—C1	120.6 (3)	O3—C17—H17B	110.3
C5—C6—H6	119.7	C18—C17—H17B	110.3
C1—C6—H6	119.7	H17A—C17—H17B	108.5
O4—C7—C1	125.0 (3)	C17—C18—H18A	109.5
O4—C7—H7	117.5	C17—C18—H18B	109.5
C1—C7—H7	117.5	H18A—C18—H18B	109.5
O6—C8—C9	107.6 (3)	C17—C18—H18C	109.5
O6—C8—H8A	110.2	H18A—C18—H18C	109.5
C9—C8—H8A	110.2	H18B—C18—H18C	109.5

Symmetry codes: (i) −*x*, −*y*+1, −*z*; (ii) −*x*, −*y*, −*z*.
